# Insulin Topical Application for Wound Healing in Nondiabetic Patients

**DOI:** 10.1155/2021/9785466

**Published:** 2021-11-18

**Authors:** Shudong Sun, Lei Zhang, Jun Liu, Huiling Li

**Affiliations:** ^1^Department of Burn and Wound Repair, Weifang People's Hospital, Weifang, Shandong, China; ^2^Department of Burns and Plastic Surgery, Binzhou People's Hospital Binzhou, Shandong, China; ^3^Department of Dermatology, Sunshine Union Hospital, Weifang, Shandong, China; ^4^Department of Burn and Wound Repair Weifang People's Hospital, Weifang, Shandong, China

## Abstract

**Background:**

Low-cost and safe strategies to improve wound healing will be of great social and economic value. The goal of this pilot clinical trial is aimed at analyzing how effective insulin therapy is at healing wounds in nondiabetic people.

**Methods:**

In this protocol research, 346 individuals were included. Patients were divided as 2 groups at random: experimental patients were given a ten-unit answer. For each 10 cm^2^ of wound, insulin was injected in solution with 1 mL 0.9 percent saline, whereas the control group got a standard dressing with normal saline.

**Results:**

During the therapy period, no adverse effects were reported. After insulin therapy, no substantial insulin-related side effects were reduced. After 10 days of therapy, the experimental group's granulation tissue coverage rate and thickness were considerably improved as compared to control. Furthermore, a momentous difference in the occurrence of wound bleeding and suppurative wounds between the two groups (*P* = 0.05).

**Conclusion:**

The results of this pilot research suggest that insulin injections could harmless and effective alternative therapy for wound healing in nondiabetic individuals and that larger, placebo-controlled trials are needed to evaluate effectiveness and safety of insulin treatment in wound healing patients.

## 1. Introduction

Hemostasis, epithelization, angiogenesis, granulation tissue development, and collagen deposition were the different stages in the wound healing process [1]. Chronic wounds afflict roughly 6.5 million peoples in the US, and over $25 billion were wasted in its care for each year. It also has a significant impact on people's quality of life [2]. As a result, successful wound healing treatments will have a significant societal impact.

Biologically insulin is a hormone (peptide) and GF (growth factor) that has been shown in previous research to help restore damaged skin [3, 4]. Insulin has been shown by Hrynyk et.al to aid in the early recovery of burn wounds [5]. Insulin increases the growth and development of several cell types, as well as keratinocytes, endothelial cells, and fibroblasts' proliferation, migration, and secretion [6]. Furthermore, topical insulin treatment for wound healing produced fewer side effects (such as hypoglycemia) and was less expensive. Although growth factors and stem cells have shown efficacy in promoting wound healing, these therapies are highly expensive and their safety remains to be evaluated. Therefore, low-cost and safe strategies to improve wound healing will be of great social and economic value.

Although many studies have addressed the healing effect of systemic insulin on burn wounds, only a few have investigated the efficacy of topical insulin. Therefore, this study is aimed at reviewing how topical insulin affected granulation tissue development and wound healing in nondiabetic individuals.

## 2. Method

### 2.1. Study Design

This was a research experiment that looked at efficacy in using insulin (topical) for wound healing among nondiabetic people. 346 patients with skin wounds attending Weifang People's Hospital and Binzhou People's Hospital were enrolled in the study, setting in the period from January 2016 to January 2020.

The procedures of this clinical trial are presented Figure 1. All patients had their complete medical history documented, including the origin, start, duration, length of wound(s), any current conservatory or complication, smoking, and any prior or current medicines that might impact the healing process (Table 1).

### 2.2. Inclusion Criteria

The inclusion criteria are as follows: (1) acute wounds (burns or crush wounds) and (2) age ≤ 75 years old.

### 2.3. Exclusion Criteria

The exclusion criteria are as follows: (1) age > 75 years old or diabetes mellitus; (2) pregnancy; (3) patients with blood systemic illnesses; and (4) patients with blood systemic diseases (immunosuppressive treatment was administered to the patients); (5) wounds that are complicated (e.g., bleeding or infection); (6) medications that may impact the study's outcome; (7) cardiovascular illnesses; (8) peripheral artery disease; and (9) renal and hepatic failure.

### 2.4. Ethics

The Ethical Committees of Weifang People's Hospital and Binzhou People's Hospital authorised this clinical trial, and all subjects gave written informed permission. This study followed the Declaration of Helsinki's recommendations.

### 2.5. Preparation

All wounds were thoroughly cleansed with physiologic serum before the therapeutic treatment began (i.e., saline 0.9 percent). A surgical blade (bistori) and local anaesthetic were used to debride dirty or crusty wounds. Sterile gauze packing was used to reduce postdebridement haemorrhage. Meanwhile, we measure the length of the wound and confirm that there is no active bleeding and exposure of important blood vessels, nerves, and tendons.

### 2.6. Treatment

The 316 individuals who were eligible for this research were randomly assigned to one of two groups: insulin (*n* = 158) or control (*n* = 158).

For each 10 cm^2^ of wound, patients in the experimental group got ten units (0.1 mL) of insulin crystal (Novo Nordisk Medicine Co., Ltd.) in solution with 1 mL saline (0.9 percent). An insulin syringe needle was used to spray the solution twice daily on the wound area. For every 10 cm^2^ of wound in the control group, 1 mL 0.9 percent saline was given. In all groups, the topical therapy was given twice a day, permitted to dry for half an hour, and covered in sterile cotton gauze. Patients were placed in such a way as to avoid solution run-off from the wound. Treatment groups and strategies for guaranteeing blindness were not disclosed to either the patient or the physician. The participants agreed to get treatment in stages until their wounds healed.

Surgically, the necrotic tissue (dead) adhering to incision was debrided. Before applying dressing, all of the wounds were carefully cleaned with 0.9 percent normal saline. Antibiotics were administered systemically based on the culture of pus and sensitivity. In a dressing process, the wound was examined towards granulation tissue, wound discharge, and infection control. The difference between two groups was assessed as a decrease in wound size.

### 2.7. Assessment of Efficacy of Insulin Therapy

The major goal of this study was to achieve complete wound closure. The main area − final wound area (in mm^2^)/healing time (in days) was used to determine the wound healing rate, which was reported as mm^2^/day [7]. When a wound was entirely closed and epithelialized, it was termed fully healed. We also look at the pace of granulation tissue covering and the thickness of granulation tissue to see how wound healing is progressing.

The primary end point was safety and adverse effect. General adverse effects were recorded as headache, palpitation, and vertigo (due to hypoglycemia); meanwhile, in both groups, glucose levels in blood were deliberated using a glucometer 10 minutes prior and 60 minutes afterwards topical drug administration. During follow-up, all adverse events were recorded and reviewed by an impartial committee.

### 2.8. Statistical Analysis

The mean ± SD was used to express all study findings. The statistical significance between the groups was determined using the *t*-test. A statistically significant *P* value of 0.05 was used. The statistical analysis was performed using SPSS 22.0 software (SPSS Inc., Chicago, IL, USA).

## 3. Results

### 3.1. The Subjects' Characteristics

Thirteen among the 338 nondiabetic patients enrolled did not satisfy the inclusion criteria, and nine were unwilling to participate in the study. Finally, 316 suitable patients were included in this pilot research, and they were randomly assigned to one of two groups: insulin (158 patients) or control (158 patients) (Figure 1). During the study, 12 patients from the experimental group were removed, whereas 8 patients from the control group were removed. Finally, 146 samples in the experimental team and 150 patients in control were examined. Table 1 shows the demographic features of the subjects. The means of age, weight, BMI, size of the wound, healing rate, and time to healing of the experimental group were 47.4 ± 5.27 years, 66.4 ± 8.96 kg, 22.73 ± 1.39 kg/m^2^, 313.53 ± 147.24 cm^2^, 46.7 ± 19.52 mm^2^/day, and 34.4 ± 10.24 days, respectively, while those of the control group were 45.4 ± 5.46 years, 61.53 ± 7.96 kg, 21.87 ± 1.86 kg/m^2^, 279.56 ± 105.15 cm^2^, 30.47 ± 14.10 mm^2^/day and 32.7 ± 9.38 days, respectively. As shown in Table 1, there is no noteworthy distinction in the age, weight, BMI, size of the wound, wound classification, and time to healing between two groups (*P* > 0.05). Surprisingly, the experimental group's healing rate was considerably higher (*P* < 0.05).

### 3.2. Therapy of Safety Evaluation

During the course of our study, no adverse events were recorded. Hypoglycemia, sweating, palpitations, and headaches were not reported as a result of insulin absorption through the incision. There were no significant side effects, such as allergic reactions or fever.

### 3.3. Clinical Efficacy of Therapy

After insulin therapy, patients' clinical wound healing rates improved. The rate of wound healing improved substantially (*P* = 0.008). (Table 1). Furthermore, we recorded the progress of wound healing of one patient who received insulin treatment (Figure 2). This showed that topical wound insulin injection had a clear influence on granulation tissue development. On day 20 following injection, the insulin group had greater granulation tissue development and wound closure, as illustrated in Figure 2.  Table 2 shows that after 10 days of therapy, the experimental group's granulation tissue coverage rate and thickness were 32.610.1 percent and 3.470.84 mm, respectively, which were substantially better compared to the control (*P* < 0.05). (Table 3); the occurrence of bleeding of wound and suppurative wounds between two groups had significant difference (6.8% vs. 10.7%, 1.4% vs. 5.3%, *P* < 0.05). And the occurrence of other complications (such as wound infection, malnutrition, hypoproteinemia, osteomyelitis, and septicemia) had no observable discernible disparity between two groups (*P* > 0.05).

## 4. Discussion

The coverage, healing rate, and thickness of granulation tissue were all enhanced in this pilot study, which exhibited that the topical insulin injection might increase wound healing among nondiabetic individuals. Furthermore, the findings of this protocol study revealed that no major adverse events occurred during the study period, indicating that topical insulin therapy in nondiabetic patients is safe.

Previous researchers have found that topical treatments have a therapeutic impact on wounds [8–14], which supports the current findings. In control and positive control animals, insulin solution administration (BD for fortnight) improved the target activity through reducing the duration of epithelialization [15]. Although wound care and management have a long history in China, wound healing research and management have made significant progress only in recent years. In diabetic rats with dry eye syndrome, it was reported that insulin-loaded microparticulate (50 L, 1 IU/mL insulin) administered every day for 15 days restored fluid volume of tear, thickness of cornea, and preserved morphology of corneal cell [8]. In a phase I study, researchers evaluated the effectiveness of topical regular crystalline insulin (including zinc), solution of aq. zinc chloride, and saline in healing open, simple cutaneous wounds and found that insulin was more effective than aqueous zinc solution [7]. As a result, research into the underlying processes of therapy of insulin for target action has exploded around recent years.

Topical preparation enhances wound healing via minimizing oxidative and inflammatory responses [16–20]. In rats with burn wounds, topical insulin therapy reduces ROS; it shall have negative action on lipids, proteins, and DNA [17]. Another research found that topical insulin causes early neutrophil recruitment and has an anti-inflammatory impact in wounds by raising IL-10 levels, which helps in removing dead tissues [18]. Similarly, topical administration of insulin to skin lesions stimulates keratinocyte migration, speeds reepithelialization, and boosts fibroblastic response, and it was carried out by the PI3K-AktRac1 pathway [17]. Increases in coverage rate, thickness of granulation tissue, and rate of wound healing were detected following insulin treatment in this investigation, which is consistent with the previous findings. Despite this, due to a lack of cytokine profiles, we are unable to determine the therapeutic mechanism of insulin. Local therapy with insulin for healing of wound among nondiabetic individuals appears to be a hopeful therapeutic option.

Furthermore, we demonstrated that insulin through topical route could safe and does not influence blood glucose levels, as well as its use in wound healing among nondiabetic individuals. Furthermore, there is no momentous dissimilarity in the occurrence of other complications (such as wound infection, malnutrition, hypoproteinemia, osteomyelitis, and septicemia) among 2 groups (*P* > 0.05), and there are no considerable ADRs of absorption of insulin from wound, like hypoglycemia, sweating, palpitations, or headache. Last but not least, future research into the physiologic pathways through which insulin aids normal wound healing is yet completely unexplored.

## 5. Conclusion

Insulin injections may be a safe and practical wound healing treatment in nondiabetic individuals, according to this protocol clinical research. To further investigate usefulness and wellbeing of insulin therapy for wound healing patients, bigger, placebo-controlled, multicenter trials are required.

## Figures and Tables

**Figure 1:** Flow chart showing recruitment.

**Figure 2:** An examination of a patient's wound in the insulin therapy group. The patient was a 56-year-old man. His left hand was lacerated (a). Following the debridement of necrotic tissue, there appeared an incision on the palm of the left hand. The granulation tissue developed nicely, and the lesion fully closed after 20 days of local insulin infusion (b).

**Table 1:** Clinical features of patients with wounds in the experimental and control groups.

	Experimental group (*n* = 146)	Control group (*n* = 150)	*t*	*P* value
Age (years)	47.4 ± 5.27	45.4 ± 5.46	0.35	0.213
Female	63 (43.2%)	88 (58.7%)	—	—
Male	83 (56.8%)	62 (41.3%)	—	—
Weight (kg)	66.4 ± 8.96	61.53 ± 7.96	0.24	0.576
BMI (kg/m^2^)	22.73 ± 1.39	21.87 ± 1.86	0.28	0.18
Size of the wound (cm^2^)	313.53 ± 147.24	279.56 ± 105.15	0.67	0.59
Area of the body affected				
Upper extremity	48 (32.9%)	53 (35.3%)	—	—
Lower limb	57 (39%)	45 (30%)	—	—
Back	11 (7.5%)	14 (9.3%)	—	—
Face	3 (2%)	5 (3.3%)	—	—
Anterior thorax	9 (6.2%)	10 (6.7%)	—	—
Abdomen	12 (8.2%)	13 (8.7%)	—	—
Sacrum	2 (1.4%)	4 (2.7%)	—	—
Head	4 (2.7%)	6 (4%)	—	—
Cause of the wound				
Trauma	79 (54.1%)	94 (62.7%)	—	—
Burn	10 (6.8%)	13 (8.7%)	—	—
Pressure	33 (22.6%)	29 (19.3%)	—	—
Scald	24 (16.4%)	14 (9.3%)	—	—
Wound classification				
Clean	40 (27.4%)	37 (24.7%)		
Clean contaminated	32 (21.9%)	39 (26%)		
Contaminated	39 (26.7%)	42 (28%)		
Dirty	35 (24.4%)	32 (21.3%)		
Healing rate (mm^2^/day)	46.7 ± 19.52	30.47 ± 14.100.91		0.008^∗^
Time to healing (days)	34.4 ± 14.24	32.7 ± 9.381.44		0.39

Note: significant difference as *P* < 0.05.

**Table 2:** After 10 days of therapy, the development of granulation tissue in the two groups was compared.

	Experimental group (*n* = 146)	Control group (*n* = 150)	*t*	*P* value
Granulation tissue coverage rate (%)	32.6 ± 10.1	21.4 ± 8.9	10.78	<0.05^∗^
The thickness of granulation tissue (mm)	3.47 ± 0.84	2.60 ± 1.92	25.37	<0.05^∗^

Note: significant difference as *P* < 0.05.

**Table 3:** After therapy, complications in the two groups were compared.

	Experimental group (*n* = 146)	Control group (*n* = 150)	*t*	*P* value
Bleeding of wound (%)	10 (6.8%)	16 (10.7%)	5.843	0.041^∗^
Wound infection (%)	6 (4.1%)	11 (7.3%)	4.931	0.054
Suppurative wounds	2 (1.4%)	8 (5.3%)	6.172	0.045^∗^
Malnutrition	8 (5.5%)	16 (10.7%)	5.624	0.059
Hypoproteinemia	9 (6.2%)	15 (10%)	5.361	0.054
Osteomyelitis	1 (0.7%)	4 (2.7%)	3.128	0.143
Septicemia	3 (2.1%)	7 (4.7%)	2.195	0.642

Note: significant difference as *P* < 0.05.

## Data Availability

The data used to support this study are available from the corresponding author upon request.

## Abbreviations

IL-10: Interleukin-10
PI3K/Akt pathway: Phosphoinositide 3-kinase/protein kinase B pathway.
